# MicroRNA-221 promotes cell proliferation, migration, and differentiation by regulation of ZFPM2 in osteoblasts

**DOI:** 10.1590/1414-431X20187574

**Published:** 2018-10-18

**Authors:** Xingguo Zheng, Jinhua Dai, Haijun Zhang, Zhibin Ge

**Affiliations:** 1 Department of Orthopaedics, Ningbo No. 2 Hospital, Ningbo, China; 2 Department of Clinical Laboratory, Ningbo No. 2 Hospital, Ningbo, China

**Keywords:** MicroRNA-221, Bone fracture, Osteoblast differentiation, ZFPM2, Wnt/Notch, Smad

## Abstract

Bone fracture is a common medical condition, which may occur due to traumatic injury or disease-related conditions. Evidence suggests that microRNAs (miRNAs) can regulate osteoblast differentiation and function. In this study, we explored the effects and mechanism of miR-221 on the growth and migration of osteoblasts using MC3T3-E1 cells. The expression levels of miR-221 in the different groups were measured by qRT-PCR. Then, miR-221 mimic and inhibitor were transfected into MC3T3-E1 cells, and cell viability and migration were measured using the CCK-8 assay and the Transwell migration assay. Additionally, the expression levels of differentiation-related factors (*Runx2* and *Ocn*) and *ZFPM2* were measured by qRT-PCR. Western blot was used to measure the expression of cell cycle-related proteins, epithelial-mesenchymal transition (EMT)-related proteins, ZFPM2, and Wnt/Notch, and Smad signaling pathway proteins. miR-221 was significantly up-regulated in the patients with lumbar compression fracture (LCM) and trochanteric fracture (TF). miR-221 promoted ALP, Runx2, and OPN expressions in MC3T3-E1 cells. miR-221 overexpression significantly increased cell proliferation, migration, differentiation, and matrix mineralization, whereas suppression of miR-221 reversed these effects. Additionally, the results displayed that *ZFPM2* was a direct target gene of miR-221, and overexpression of ZFPM2 reversed the promoting effects of miR-221 overexpression on osteoblasts. Mechanistic study revealed that overexpression of miR-221 inactivated the Wnt/Notch and Smad signaling pathways by regulating ZFPM2 expression. We drew the conclusions that miR-221 overexpression promoted osteoblast proliferation, migration, and differentiation by regulation of ZFPM2 expression and deactivating the Wnt/Notch and Smad signaling pathways.

## Introduction

Bone fracture is a common and increasing disease, which results from both traumatic injury and disease-related bone fragility (1). In the United States, about six million adults suffer from fractures annually (2). Bone fracture may lead to fever, disability, shock, and treatment is very expensive. Timely and appropriate management of bone fractures can help patients restore original functions. However, some patients still have different degrees of sequelae, such as osteomyelitis, non-union and mal-union, complex regional pain syndrome, and post-traumatic arthritis (3). Bone fracture healing is a physiologically complex process, which involves both biological and mechanical factors (4). Following bone fracture, a series of events occurs, including cell migration, differentiation, tissue synthesis, and the release of cytokines and growth factors. The recovery process of fracture depends on the activity of osteoblasts (5,6). Osteoblasts are mesenchymal cells, which play a major role in skeletal development and bone formation (7). Osteoblasts are responsible for the synthesis, secretion and mineralization of bone matrix (8). Therefore, it is necessary to explore the mechanism of osteoblast proliferation, migration, and differentiation.

MicroRNAs (miRNAs) are small, non-coding RNA molecules, which can mediate the post-transcriptional gene expression (9). A recent study demonstrates that miRNAs are involved in various cellular processes, such as cell proliferation, migration, differentiation, and apoptosis (10). Increasing evidence indicates that miRNAs regulate the differentiation and function of chondrocytes, osteoblasts, and osteoclasts (11). These findings suggest that miRNAs act as key mediators in the processes of bone formation, resorption, remodeling, and repair (12). As Waki et al. (13) reported, several miRNAs, such as miR-140-3p, miR-140-5p, miR-181a-5p, miR-181d-5p, and miR-451a, were significantly up-regulated in standard healing fractures compared with unhealing fractures. Moreover, more than 15 miRNAs have been reported for bone formation stimulation (14). miR-221 is one of many widely studied miRNAs, which is frequently up-regulated in various cancers (15,16). However, the precise function of miR-221 in bone fracture is still unknown. In this study, we aimed to explore the role of miR-221 in osteoblast proliferation, migration, and differentiation using MC3T3-E1 cells. This is the first study to report the effects of miR-221 on osteoblast growth and differentiation in the bone fracture healing process. This study might provide novel therapeutic strategies for bone fracture.

## Material and Methods

### Blood sample collection

The blood samples were obtained from three patients with lumbar compression fracture (LCM) and three patients with trochanteric fracture (TF) of Ningbo No.2 Hospital from April 2017 to October 2017. The blood samples were collected at 24 h and 7, 14, and 21 days after surgery or injury and then stored at –80°C until analyzed. The ethical approval for this study was granted by the Ethics Committee of Ningbo No. 2 Hospital. All participants signed the informed consent.

### Cell culture and differentiation induction

The mouse osteoblast-like cells (MC3T3-E1) used in the present study were obtained from American Type Culture Collection (ATCC, USA). The cells were cultured in 100-mm dishes containing α-MEM culture medium with 10% fetal bovine serum (FBS, Gibco, USA), and 1% penicillin and streptomycin under humid environment with 5% CO_2_ at 37°C. The culture medium was changed every three days. For induction of MC3T3-E1 cells differentiation, 1×10^5^ cells were seeded in a 6-well plate, and incubated in the differentiation medium containing 50 µg/mL ascorbic acid and 10 mmol/L β-glycerophosphate. The control group cells were cultured with conventional medium. The medium was refreshed every three days.

### Quantitative real-time polymerase chain reaction (qRT-PCR) analysis

Total RNA was isolated from blood samples using the PAXgene Blood RNA Kit (Qiagen, Germany) and from MC3T3-E1 cells using the common kit of Trizol reagent (Invitrogen, Life Technologies Corporation, USA) according to manufacturer's protocols. For examining the expression level of miR-221 in MC3T3-E1 cells, cDNA was synthesized using TaqMan MicroRNA Reverse Transcription Kit (Invitrogen), and qRT-PCR analysis was carried out using TaqMan Universal Master Mix II (Invitrogen) following the instructions, and U6 (Applied Biosystems, USA) was used to normalized the expression level of miR-221. Data were examined by the 2^-ΔΔCt^ method.

### miRNAs transfection

The expression plasmids of miR-221 mimic, miR-221 inhibitor, and the corresponding negative controls (NCs) were synthesized by GenePharma Co. (China). Additionally, the overexpression vector of zinc finger protein multitype 2 (ZFPM2) was constructed using the sub-cloning the full-length ZFPM2 coding sequence into pcDNA3.1 plasmid (Sangon Biotech, China). The empty pcDNA3.1 plasmid was used as a negative control. Afterward, MC3T3-E1 cells were transfected with these expression plasmids for 48 h. All cell transfections were detected using Lipofectamine 3000 reagent (Invitrogen) according to the manufacturer's protocol.

### Cell viability assay

Cell viability of MC3T3-E1 cells was detected using the Cell Counting Kit-8 (CCK-8) assay (Beyotime Biotechnology, China). Briefly, MC3T3-E1 cells were cultured in a 96-well plate, and transfected with expression vectors of miR-221 mimic, miR-221 inhibitor, and pc-ZFPM2. After transfection for 48 h, 10 μL CCK-8 was supplemented to each well and the plates were incubated for another 1 h under the routine-culture environment containing 95% air and 5% CO_2_ at 37°C. Finally, a microplate reader (Bio-Rad, USA) was used to measure the absorbance at 450 nm.

### Cell migration assay

For the migration assay, the Transwell with a pore size of 8 μM was performed to examine the migration ability of MC3T3-E1 cells. In brief, MC3T3-E1 cells were transfected with the above expression vectors. Afterward, these cells were suspended in serum-free medium, and 100-μL cell suspension was added into the upper compartment of a 24-well transwell culture chamber. Meanwhile, 600 μL of complete medium was added into the lower compartment. After incubation for 24 h in the conventional culture conditions, the Transwell culture chamber was taken out, and washed twice with calcium-free PBS, and cells were fixed with methanol for 30 min. Subsequently, the non-migrated cells were removed carefully using a wet cotton swab from the upper surface of the filter. The migrated cells on the lower side of the filter were stained with 1% crystal violet for 20 min, and counted using a microscope (magnification of 400×) in a random five fields of vision.

### Alizarin Red S staining assay

To confirm the important effects of miR-221 on mineralization of MC3T3-E1 cells, the Alizarin Red S staining assay was performed. Briefly, the cells were washed twice with PBS and fixed with 95% ethanol for 10 min at room temperature. Subsequently, the fixed cells were stained with 1% Alizarin Red S solution (Sigma-Aldrich, USA) for 30 min at 37°C and counted using a light microscope (Olympus, Japan). Quantification of Alizarin Red S stain was assessed via extraction with Image J software (NIH, USA).

### Luciferase reporter assay

The 3′-untranslated region (3′-UTR) of ZFPM2 was amplified by PCR and inserted into pmiR-Report vector (Promega, USA). Then, the vectors were co-transfected with miR-221 mimic and its corresponding control into cells using Lipofectamine 3000 (Invitrogen). The luciferase assay was confirmed using the dual luciferase reporter assay system (Promega) after transfection for 48 h.

### Western blot assay

The proteins from transfected cells used for the western blot assay were isolated using RIPA lysis buffer (Beyotime Biotechnology). The contents of total protein were tested using the BCA™ Protein Assay Kit (Pierce, USA) based on the kit instruction. Then, 40 μg protein samples were subjected to sodium dodecyl sulfate-polyacrylamide gel electrophoresis (SDS-PAGE) and transferred to polyvinylidene difluoride (PVDF) membranes. After blocking with 5% non-fat milk, the membranes were transferred to another container and incubated with the primary antibodies of alkaline phosphatase (ALP, ab83259), Runt-related transcription factor 2 (Runx2, ab23981), Osteopontin (OPN, ab8448), E-cadherin (ab40772), N-cadherin (ab18203), Vimentin (ab16700), ZEB1 (ab124512), Snail (ab82846), Osteocalcin (Ocn, ab93876), proliferating cell nuclear antigen (PCNA, ab18197), Cyclin A (ab181591), Cyclin E1 (ab71535), cyclin-dependent kinase 2 (CDK2, ab64669), Cyclin D1 (ab134175), CDK4 (ab199728), Wnt3a (ab28472), Wnt5a (ab229200), Notch 1 (ab52627), Notch 2 (ab8926), Notch 3 (ab23426), p-Smad2 (ab53100), Smad2 (ab33875), Smad4 (ab40759), Smad7 (ab216428), and GAPDH (ab181602) at 4°C overnight. After incubation for 2 h at 37°C, the secondary antibody of horseradish peroxidase (HRP)-conjugated goat anti-rabbit IgG (ab205718, 1:2000, Abcam) was added and incubated for 1 h at room temperature. Finally, the signals were captured using ECL reagents (MultiSciences Biotech, China).

### Statistical analysis

The results are reported as means±SD. SPSS 19.0 statistical software (SPSS, Inc., USA) was used to analyze the data. One-way analysis of variance (ANOVA) was used to calculate the P values. P<0.05 was considered to be statistically significant.

## Results

### miR-221 was up-regulated during osteoblast differentiation

To explore the effect of miR-221 on bone fracture, the blood concentrations of miR-221 in three LCM patients and three TF patients were examined. The results showed that the blood concentrations of miR-221 were obviously increased at 7 and 14 days after surgery, whereas the concentrations of miR-221 was recovered at 21 days after surgery (Figure 1A and B). Additionally, MC3T3-E1 cells were cultured in osteogenic differentiation medium, and the relative expression of miR-221 during the osteoblast differentiation process was detected at different time intervals (0, 4, 7, 14, 21, and 28 days) using qRT-PCR. As shown in Figure 1C, the expression of miR-221 was significantly increased in a time-dependent manner during osteoblastic differentiation. Further, the western blot assay revealed that the protein levels of ALP, Runx2, and OPN were notably up-regulated in a time-dependent manner (P<0.001, Figure 1D and E). These data indicated that up-regulation of miR-221 might have an important role in the process of bone fracture.

**Figure 1.** miR-221 is up-regulated during the osteoblast differentiation process. *A* and *B*, Blood concentrations of miR-221 in three lumbar compression fracture (LCM) patients and three trochanteric fracture (TF) patients were examined by qRT-PCR. Then, MC3T3-E1 cells were treated with osteogenic differentiation media. *C*, Expression of miR-221 during osteoblast differentiation at 0, 4, 7, 14, 21, and 28 days was detected by qRT-PCR. *D* and *E*, Protein levels of ALP, Runx2, and OPN were assessed by western blot. *miR*-221: microRNA-221; qRT-PCR: quantitative reverse transcription polymerase chain reaction; ALP: alkaline phosphatase; Runx2: runt-related transcription factor 2; OPN: osteopontin. Data are reported as means±SD. ***P<0.001 compared to baseline (ANOVA).

### Overexpression of miR-221 promoted osteoblast proliferation

Next, MC3T3-E1 cells were transfected with miR-221 mimic, miR-221 inhibitor, and the corresponding controls. After transfection for 48 h, the expression level of miR-221 was measured using qRT-PCR. The results in Figure 2A showed that miR-221 overexpression significantly increased the expression of miR-221 compared with the mimic control group (P<0.01), while miR-221 suppression significantly decreased the expression of miR-221 compared with the inhibitor control group (P<0.001). We then measured cell viability using the CCK-8 assay. As shown in Figure 2B, miR-221 overexpression significantly promoted cell viability compared with the mimic control group (P<0.05), whereas miR-221 suppression significantly decreased cell viability compared with the inhibitor control group (P<0.05). Western blot assay was performed to further confirm these results by analysis of cell cycle-related proteins (PCNA, Cyclin A, Cyclin E1, CDK2, Cyclin D1, and CDK4). The results showed that miR-221 overexpression increased the expression of these proteins, whereas miR-221 inhibition decreased their expression in MC3T3-E1 cells (P<0.01, Figure 2C and D). Taken together, the data indicated that overexpression of miR-221 could promote cell proliferation.

**Figure 2.** Overexpression of miR-221 promoted osteoblast proliferation. *A*, Expression of miR-221 in transfection of MC3T3-E1 cells was detected using qRT-PCR. *B*, Cell viability was measured using the CCK-8 assay. *C* and *D*, Western blot was used to measure the expression of cell cycle-related proteins. miR-221: microRNA-221; qRT-PCR: quantitative reverse transcription polymerase chain reaction; CCK-8: cell counting kit-8; PCNA: proliferating cell nuclear antigen; CDK: cyclin-dependent kinase; qRT-PCR: quantitative reverse transcription polymerase chain reaction. Data are reported as means±SD. *P<0.05, **P<0.01, ***P<0.001 (ANOVA). NS: not significant.

### Overexpression of miR-221 promoted osteoblast migration

The results of the Transwell migration assay showed that miR-221 overexpression remarkably increased cell migration compared with the mimic control group (P<0.05), whereas miR-221 suppression significantly decreased cell migration compared with the inhibitor control group (P<0.05, Figure 3A). Western blot results showed that miR-221 overexpression decreased the expression of E-cadherin (P<0.01), as well as increased the expressions of N-cadherin, Vimentin, ZEB1, and Snail (P<0.01). However, miR-221 suppression showed opposite results (Figure 3B and C). These findings indicated that overexpression of miR-221 could promote cell migration and EMT process in osteoblasts.

**Figure 3.** Overexpression of miR-221 promotes osteoblast migration. *A*, Cell migration was measured using the Transwell migration assay. *B* and *C*, Protein levels of EMT-related proteins (E-cadherin, N-cadherin, Vimentin, ZEB1, and Snail) were determined using western blot. miR-221: microRNA-221; EMT: epithelial-mesenchymal transition. Data are reported as means±SD. *P<0.05, **P<0.01 (ANOVA).

### Overexpression of miR-221 promoted osteoblast differentiation

qRT-PCR results of cell differentiation showed that miR-221 overexpression significantly increased the expression of Runx2 and Ocn on days 7 and 14, whereas miR-221 suppression showed opposite results (P<0.05, Figure 4A and B). Mineralization analysis showed that overexpression of miR-221 significantly increased the mineralized nodule formation compared with the control group (P<0.01, Figure 4C). Furthermore, the results of western blot (Figure 4D-F) revealed that miR-221 overexpression notably increased the protein levels of ALP, Runx2, and Ocn on days 7 and 14, whereas miR-221 suppression showed opposite results except for Ocn expression on day 14, which was unchanged. Above all, the results suggested that overexpression of miR-221 was associated with osteoblast differentiation.

**Figure 4.** Overexpression of miR-221 promoted osteoblast differentiation. The mRNA expressions of (*A*) Runx2 and (*B*) Ocn were measured using qRT-PCR. *C*, The mineralized nodule formation in MC3T3-E1 cells with miR-221 overexpression was examined using the Alizarin Red S staining assay. *D-F*, Protein levels of ALP, Runx2, and Ocn were determined by western blot. miR-221: microRNA-221; ALP: alkaline phosphatase; Runx2: runt-related transcription factor 2; Ocn: osteocalcin; qRT-PCR: quantitative reverse transcription polymerase chain reaction. Data are reported as means±SD.*P<0.05, **P<0.01, ***P<0.001 (ANOVA).

### ZFPM2 was a direct target of miR-221

To explore the relationship between miR-221 and ZFPM2, the software programs of TargetScan (http:/www.targetscan.org) and microRNA database (http:/www.microrna.org) were used to predict the binding site (Figure 5A). Then, the expression level of ZFPM2 in MC3T3-E1 cells transfected with miR-221 mimic and miR-221 inhibitor was detected by qRT-PCR and western blot. The results showed that the mRNA and protein levels of ZFPM2 were significantly decreased by miR-221 overexpression, as well as promoted by miR-221 suppression (P<0.05, Figure 5B). Meanwhile, dual-luciferase reporter assay results showed that luciferase activity was greatly decreased by co-transfection of miR-221 mimic and ZFPM2-WT (P<0.05). However, co-transfection of miR-221 mimic and ZFPM2-MUT had no effect on luciferase activity (Figure 5C). In short, the results indicated that ZFPM2 was a direct target gene of miR-221, and miR-221 inhibited ZFPM2 expression in osteoblasts.

**Figure 5.** ZFPM2 was a direct target of miR-221. *A*, The binding site of miR-221 and ZFPM2 was analyzed by TargetScan and microRNA database. *B*, mRNA and protein levels of ZFPM2 were examined by qRT-PCR and western blot. *C*, The relationship between miR-221 and ZFPM2 was detected by dual-luciferase reporter assay. ZFPM2: zinc finger protein multitype 2; miR-221: microRNA-221; qRT-PCR: quantitative reverse transcription polymerase chain reaction. Data are reported as means±SD. *P<0.05 (ANOVA).

### Overexpression of miR-221 promoted osteoblast proliferation, migration, and differentiation by targeting ZFPM2

To uncover whether ZFPM2 was involved in the processes of osteoblast proliferation, migration, and differentiation, miR-221 mimic and pc-ZFPM2 were transfected into MC3T3-E1 cells to change miR-221 and ZFPM2 expression. The results in Figure 6A and B showed that miR-221 overexpression significantly increased cell viability and migration compared with the mimic control group (P<0.05), but overexpression of ZFPM2 reversed these effects by decreasing cell viability and migration (P<0.05). Western blot results revealed that overexpression of miR-221 increased the expression of cell cycle-related proteins (PCNA, Cyclin A, Cyclin E1, CDK2, Cyclin D1, and CDK4), but overexpression of ZFPM2 reversed these effects (P<0.05, Figure 6C and D). Moreover, the expression level of differentiation-related proteins (ALP, Runx2, and Ocn) were increased by miR-221 mimic, but overexpression of ZFPM2 reversed these effects (P<0.05, Figure 6E and F). These findings indicated that overexpression of miR-221 promoted cell viability, migration, and differentiation by regulating the expression of ZFPM2.

**Figure 6.** Overexpression of miR-221 promotes osteoblast viability, migration, and differentiation by regulation of ZFPM2. *A*, Cell viability was measured using the CCK-8 assay. *B*, Cell migration was measured using the Transwell migration assay. *C* and *D*, Protein levels of cell cycle-related proteins were measured using western blot. *E* and *F*, Protein levels of differentiation-related proteins were detected by western blot. miR-221: microRNA-221; ZFPM2: zinc finger protein multitype 2; CCK-8: cell counting kit-8; PCNA: proliferating cell nuclear antigen; CDK: cyclin-dependent kinase; ALP: alkaline phosphatase; Runx2: runt-related transcription factor 2; Ocn: osteocalcin. Data are reported as means±SD. *P<0.05 (ANOVA). ns: not significant.

### Overexpression of miR-221 deactivated Wnt/Notch and Smad signaling pathways

Lastly, we measured the effect of miR-221 and ZFPM2 on the Wnt/Notch and Smad signaling pathways using western blot. Overexpression of miR-221 decreased the protein level of Wnt3a, Wnt5a, Notch 1, Notch 2, Notch 3, p-Smad2, Smad4, and Smad7, but overexpression of ZFPM2 reversed these effects (P<0.05 or P<0.01, Figure 7A-D). These findings indicated that overexpression of miR-221 deactivated Wnt/Notch and Smad signaling pathways by regulation of ZFPM2.

**Figure 7.** Overexpression of miR-221 deactivated Wnt/Notch and Smad signaling pathways. MC3T3-E1 cells were transfected with mimic control, miR-221 mimic, or miR-221mimic+pc-ZFPM2. The protein levels of (*A* and *B*) Wnt3a, Wnt5a, Notch 1, Notch 2, and Notch 3, and (*C* and *D*) Smad2, Smad4, and Smad7 were determined using western blot. miR-221: microRNA-221; zFPM2: Zinc finger protein multitype 2. Data are reported as means±SD. *P<0.05, **P<0.01 (ANOVA).

## Discussion

Bone fracture is a common medical condition, which is damage in the continuity of the bone, and this disease occurs frequently in children and the elderly (17). The activity of osteoblasts is closely related to the quality of recovery of bone fractures. Osteogenesis is a complex and multistep processes, involving the differentiation of mesenchymal stem cells into osteoblast progenitor cells, preosteoblasts, osteoblasts, and osteocytes, as well as crosstalk between multiple cell types for the formation and remodeling of bone (18). The process is regulated by various signaling networks, such as BMP, Wnt ligands, Notch ligands, transforming growth factor (TGF), tumor necrosis factor, and cytokines. A recent study demonstrated that miRNAs acted as important regulators of osteogenic signaling pathways (19). In this study, we investigated the effects and mechanism of miR-221 on osteoblasts proliferation, migration, and differentiation. The results showed that miR-221 was up-regulated in the patients with LCM and TF, and closely related with the process of osteoblastic differentiation. Moreover, we found that overexpression of miR-221 significantly promoted cell proliferation, migration, differentiation, and matrix mineralization in osteoblasts, and suppression of miR-221 showed contrary results. Further experiments showed that ZFPM2 was a direct target of miR-221, and overexpression of miR-221 promoted cell viability, migration, and differentiation by down-regulation of ZFPM2. Finally, the results indicated that miR-221 overexpression blocked Wnt/Notch and Smad7 signaling pathways by regulating ZFPM2 expression.

miR-221 is one of the important miRNAs, which has been widely reported in various cancers, but it has not been fully investigated in osteoblastic differentiation (20). Several other miRNAs have been shown to be up-regulated in osteoblastic differentiation. For example, Chen et al. (21) showed that miR-34a was up-regulated in osteoblastic differentiation of human stromal stem cells. Li et al. (22) demonstrated that miR-216a was remarkably up-regulated during osteogenic differentiation in human adipose-derived MSCs. Interestingly, miR-31 was reported to be down-regulated during osteoblastic differentiation, however, miR-31 was later identified to be up-regulated during osteoblastic differentiation (23,24). Similar to these studies, we found that miR-221 was up-regulated in LCM and TF patients and also up-regulated during osteoblastic differentiation. These data indicated that miR-221 might be involved in the process of osteoblastic differentiation.

Osteogenic differentiation is divided into four stages: cellular commitment, proliferation, matrix maturation, and mineralization. Our study demonstrated that overexpression of miR-221 promoted osteoblast proliferation. In line with this finding, Xu et al. (25) showed that transfection of MC3T3-E1 osteoblasts with miR-365 ameliorated dexamethasone-induced inhibition of cell viability. Cyclins and CDKs are known to be regulators of cell cycle. An *in vitro* study has shown that Cyclin E, Cyclin B, Cyclin A, and CDK inhibitors regulate osteoblastic differentiation (26). Our study also found that overexpression of miR-221 increased the expression of cell cycle-related proteins (PCNA, Cyclin A, Cyclin E1, CDK2, Cyclin D1, and CDK4). Thus, these findings indicated that overexpression of miR-221 promoted cell proliferation in osteoblasts.

EMT is a biological process, which is characterized by a transition from epithelial cells to interstitial phenotypes by specific procedures. Mounting evidence has indicated that EMT is involved in the formation of many tissues and organs during development (27,28). Moreover, several signaling pathways, such as TGF-β, Wnt, and Notch, have been reported to induce the EMT process. These signaling pathways can activate transcription factors, including Snail, Slug, and ZEB family, which suppress the expression of E-cadherin, resulting in cell invasion and migration (29). Osteoblast migration improves the repair of bone fracture and growth of bone tissue (30). Our study found that overexpression of miR-221 promoted osteoblast migration by decreasing the expression of E-cadherin and increasing the expression of N-cadherin, Vimentin, ZEB1, and Snail.

Understanding the regulatory mechanism of osteoblast differentiation is very important to develop strategies for treating bone disorders, including bone fracture. Runx2, Osterix, and β-catenin are the vital transcription factors for osteoblast differentiation (6). Runx2 is a main transcription factor required for the differentiation of osteoblasts from mesenchymal precursors and subsequent bone matrix mineralization (31). Moreover, recent research has proven that Runx2 can directly stimulate the osteoblast marker gene expression, such as Ocn (32). Ocn is a late bone marker, which appears in osteogenic differentiation and mineralization (33). Several studies have shown the involvement of miRNAs in osteoblast differentiation. For example, miR-26a and miR-125b are shown to inhibit osteoblast differentiation, whereas miR-33-5p and miR-194 are reported to promote osteoblast differentiation (34,35). An interesting study from Zhang et al. (36) reported that miR-221 could inhibit osteogenic differentiation by targeting Runx2 in C2C12 cells. Similarly, Yeh et al. (37) found that miR-221 attenuated the osteogenic differentiation in human annulus fibrosus cells. However, the opposite results in the present study revealed that miR-221 promoted osteoblast differentiation by increasing the expression of ALP, Runx2, and Ocn in MC3T3-E1 cells. The different results might be related to the different cell lines used. Further studies are still needed to confirm the hypothesis.

ZFPM2 is a zinc finger protein encoded by the ZFPM2 gene, which is an important regulator of hematopoiesis and cardiogenesis in mammals (38). A recent study revealed that miR-429 could induce MC3T3-E1 osteoblastic cells differentiation by regulation of ZFPM2 expression (39). However, whether miR-221 affects cell proliferation, migration, and differentiation through regulating ZFPM2 expression in MC3T3-E1 cells is still unclear. In our study, we found that ZFPM2 was a direct target of miR-221. Moreover, miR-221 decreased the expression of ZFPM2 in osteoblasts. Further experiments revealed that overexpression of ZFPM2 reversed the promoting effects of miR-221 on MC3T3-E1 cells proliferation, migration, and differentiation, indicating that the effects of miR-221 on osteoblastic cells are mediated via regulating ZFPM2.

It has been reported that Wnt, Notch, and Smad signaling pathways play important roles in osteoblast differentiation (40). Therefore, we explored the effect of miR-221 and ZFPM2 on Wnt/Notch and Smad signaling pathway proteins (Wnt3a, Wnt5a, Notch 1 to 3, Smad2, Smad4, and Smad7), and found that overexpression of miR-221 decreased the protein levels of these proteins, but ZFPM2 overexpression reversed these effects, indicating that miR-221 blocked Wnt/Notch and Smad signaling pathways by regulation of ZFPM2.

In conclusion, these results revealed that miR-221 was up-regulated during osteoblastic differentiation, and overexpression of miR-221 promoted cell viability, migration, and differentiation by regulating ZFPM2 expression and deactivating the Wnt/Notch and Smad signaling pathways. Our novel findings indicate a potential role of miR-221 in osteoblast proliferation, migration, and differentiation.
